# Administration of bicarbonates through percutaneous gastrostomy with continuous nocturnal infusion in a patient with Kearns-Sayre disease: a life changing therapeutical paradigm

**DOI:** 10.1186/s13052-024-01696-9

**Published:** 2024-07-29

**Authors:** Arianna Traunero, Francesco Baldo, Andrea Magnolato, Grazia Di Leo, Egidio Barbi, Irene Bruno

**Affiliations:** 1 Department of Surgical, Medical and Health Sciences, University of Trieste, Via dell’Istria 65/1, 34127 Trieste, Italy; 2 Institute for Maternal and Child IRCCS Burlo Garofolo, Trieste, Italy

**Keywords:** Kearns-Sayre disease, Proximal renal tubular acidosis, Alkali therapy, Percutaneous endoscopic gastrostomy

## Abstract

**Background:**

Mitochondrial diseases (MDs) are systemic disorders that can affect multiple organs. Renal manifestations, including renal tubular acidosis, are common because kidneys are particularly vulnerable to energy deprivation. Treatment of MDs is often complex and electrolyte replacement can be difficult especially in pediatric patients, because large and repeated amounts of oral supplements are needed but are not well tolerated.

**Case presentation:**

We describe the case of a girl affected by Kearns-Sayre disease with severe renal tubular acidosis. The management of her metabolic acidosis was challenging because she showed persistent low levels of serum bicarbonates despite a progressive incrementation of oral bicarbonates. Furthermore, as a result to the ingestion of large amounts of alkali, the girl developed an aversion to oral supplementation. After positioning a percutaneous gastrostomy (PEG) and starting enteral administration of bicarbonates (with daily boluses and continuous nocturnal infusion), she finally obtained an adequate electrolyte control, with a significant increase in her quality of life.

**Conclusions:**

In MDs, the combination of nocturnal continuous enteral administration of alkali plus diurnal boluses may represent a valid solution to correct metabolic acidosis. It can also result in an improved patients’ quality of life, particularly in pediatric settings, where compliance to oral therapy is often lacking due to the large and repeated amounts of unpalatable bicarbonates solutions required.

## Background

Mitochondrial diseases (MDs) are complex multisystemic disorders with heterogeneous clinical presentation. They usually manifest during childhood and can affect the central nervous system and peripheral nerves, muscles (including the heart), eyes and ears, endocrine organs, lungs, gastrointestinal and urinary tract, bones, and skin. Renal involvement is often present, especially in MELAS (Mitochondrial Encephalomyopathy, Lactic Acidosis and Stroke-like episodes) syndrome, Kearns-Sayre syndrome (KSS), and mitochondrial depletion syndrome. In fact, kidney function is highly dependent on aerobic respiration, making it vulnerable to energy deprivation [1]. Defects in mitochondrial energy metabolism have been associated with various renal manifestations, involving the glomerulus, the interstice, and the tubules. As a result, nephrotic syndrome, renal tubular acidosis, Bartter-like syndrome, Fanconi syndrome, focal segmental glomerulosclerosis, tubulointerstitial nephritis, nephrocalcinosis and nephrolithiasis are all possible manifestations of kidney damage [2].

The management of MDs is usually complex and multiple treatments are often required. Electrolyte replacement may be particularly challenging because, due to renal wasting, large volumes of potassium, calcium, magnesium, phosphate, and bicarbonates supplementation may be needed. Oral assumption of large and repeated amounts of supplements may be challenging due to poor palatability, inconvenient times repeated assumptions, patient’s refusal with an insufficient intake or/and a relevant impact on quality of life.

We report on a child affected by Kearns-Sayre syndrome (KSS), a mitochondrial disease that is caused by the deletion of a variable number of base pairs of mitochondrial DNA (ranging from 1.1 to 10 kilobase). KSS reported prevalence ranges between 1 and 3 cases per 100.000 subjects. The disease is defined by the characteristic triad of external ophthalmoplegia, pigmentary retinopathy, with a typical mottled salt-and-pepper pattern of pigment clumping, and clinical onset before the age of 20. Systemic involvement includes cardiomyopathy with cardiac conduction disturbances, which can predispose to stroke and sudden death, cerebellar symptoms, progressive hearing loss which ends up in deafness, endocrine abnormalities (diabetes mellitus, growth hormone insufficiency, hypogonadotropic hypogonadism, adrenal insufficiency, primary hypoparathyroidism), non-ocular muscle weakness and renal disorders [3, 4]. The diagnosis is usually made with mitochondrial DNA analysis in peripheral blood leukocyte samples; however, in case of negative blood tests despite a strong clinical suspect, a muscle biopsy with mitochondrial DNA analysis should be performed, since tissue-specific mutations can be missed due to low levels of heteroplasmy in blood. Furthermore, skeletal muscle biopsy usually shows ragged red fibers and abnormal mitochondria. KSS treatment is exclusively supportive, and includes hormonal replacement therapy, cardiac pacemaker placement for patients with cardiac conduction blocks, cochlear implants in sensorineural hearing loss, and oral bicarbonates in renal tubular acidosis.

In this paper we will describe the case of a girl affected by KSS with severe renal tubular acidosis that required bicarbonates administration through percutaneous gastrostomy (PEG) to achieve an adequate electrolyte and pH control, with a significant increase in her quality of life.

## Case presentation

The patient was born at full term and had no perinatal problems. Developmental milestones were reached at an appropriate age. Growth was regular until the age of two, when an initial height deflection was noticed. At the age of seven, a mild right eyelid ptosis appeared, followed by asthenia, inappetence, weight loss, polyuria, and polydipsia, for which the girl was hospitalized. Blood tests highlighted a normochloremic acidosis with hypokalemia, which was explained by a Fanconi-like syndrome, characterized by proteinuria and glycosuria, with proximal renal tubular acidosis (Table 1).

**Table 1:** Blood and urinary tests at the onset of proximal tubular acidosis

Blood		Urine (spot)	
Creatinine	0.32 mg/dl	**β2 microglobuline**	**> 50,000 ng/ml**
Sodium	135 mEq/l (135–145)	Sodium	51 mEq/l
Potassium	**2.49 mEq/l (3.5–5.1)**	Potassium	27 mEq/l
Chloride	109 mEq/l (98–110)	Chloride	53 mEq/l
Calcium	9.59 mg/dl (8.5–10.5)	**Calcium/Creatinine**	**0.39 mg/g (< 0.2)**
Phosphate	**1.31 mg/dl (3.96–6.13)**	**Glucose**	**5.98 g/dl**
Bicarbonates	**19 mEq/l (22–26)**	**Proteins/Creatinine**	**4682 mg/g (< 200)**
pH	**7.35**	pH	**4.5**
Anion Gap	9.49 mEq/l	**Anion Gap**	**25 mEq/l**

To correct the electrolyte imbalance an oral supplementation with potassium phosphate and bicarbonate was started. Endocrinologic tests documented a growth hormone deficiency, as well as an adrenal insufficiency. Therefore, replacement therapy with hydrocortisone was started and was progressively increased over time (up to 10 mg/sqm/die), as well as somatropin, through which a regular growth rate was reached, although in the low percentiles per age. In the suspect of a mitochondrial disease, audiometry and ophthalmological exams were also performed, showing mild bilateral sensorineural hearing loss and corneal de-epithelialization associated with superficial neovascularization and peripheral retinal dystrophy. Muscle biopsy showed a macrodeletion of about 8000 base pairs in 40% of the mitochondrial DNA, indicative of KSS. To reduce the progressive tissue degeneration, antioxidants agents and multivitamins were also introduced in her oral therapy. Due to the worsening of the hearing impairment, hearing aids were placed with a consequent good acoustic gain.

Since the onset of the oral polytherapy, the girl’s general conditions improved. However, the management of her metabolic acidosis was challenging. In fact, despite a progressive incrementation of oral bicarbonates from 8 mEq/kg/die to 17 mEq/kg/die, blood tests showed persistent low levels of serum bicarbonates, with a median nadir value (serum concentration before the next supplementation) of 17 mEq/L HCO3- (normal range 22–26 mEq/L) and severe acidemic pH levels, reaching a minimum nadir value of 7.15. Furthermore, as a result to the ingestion of large amounts of alkali, the girl developed an aversion to bicarbonate supplementation. In fact, the only formulation of bicarbonate available was an oral solution of sodium bicarbonate, in which 1 ml of solution corresponds to 1 mEq of HCO3-. Other formulations, such as bicarbonate tablets, were impracticable for patient’s lack of compliance. The total amount of HCO3- solution administered in a day reached a dosage of 260 ml, in addition to potassium supplementations, that further increased the daily burden of treatment.

After a multidisciplinary discussion, involving nephrologists, pediatricians, and gastroenterologists, a percutaneous endoscopic gastrostomy (PEG) was placed, with the aim of obtaining a satisfactory acid-base balance with the enteral administration of the bicarbonates and other electrolytes.

The girl’s therapy was administered with the following scheme: 4 boluses of sodium bicarbonate during the day and a continuous nocturnal infusion, allowing her to take 29 mEq/kg/day of HCO3-, corresponding to a total amount of 440 mEq of solution (476 mEq of HCO3- if we also consider the amount of potassium citrate administered). This amount of alkali finally led to a normalization of the pH value, as showed in the graphic below (Table 2). The dosage was subsequently mildly modified to maintain bicarbonate levels between 22 and 24 mEq/l. In the next months the enteral nocturnal infusion was enhanced, and the daily boluses reduced in frequency (from 4 to 2 boluses), always maintaining a good acid-base balance (Table 3). Since the placement of the gastrostomy and the optimization of therapy, her quality of life has much improved: the girl was finally able to resume the daily routine as before the diagnosis, returning to school at full time, which was previously impracticable for the multiple daily therapy intake.

**Table 2:** pH and bicarbonate levels with oral alkali therapy before and after PEG placement

	Minimum nadir* values (before PEG)	Median nadir* values (before PEG)	Median values (after PEG)
pH	7.15	7.25	7.35
HCO3-	12 mEq/l	16.8 mEq/l	22.7 mEq/l

*Nadir value stands for the serum concentration of both bicarbonates and pH before the next supplementation

**Table 3:** Trend of serum bicarbonate levels before and after initiation of the enteral therapy

## Discussion and conclusions

Metabolic acidosis due to renal loss is typical of KSS and requires adequate and prompt therapy to avoid both acute metabolic decompensation (that can manifest with dyspnea, hypotension, tachycardia, nausea, vomiting, confusion, lethargy up to coma and cardiac paralysis) and chronic consequences, such as growth retardation.

Alkali administration is titrated to achieve normal serum pH and to maintain blood HCO3- levels greater than 20 to 22 mEq/l. In proximal renal tubular acidosis (pRTA), such as in KSS, the amount of bicarbonate required to achieve pH normalization may be as high as 15 mEq/kg/day. This dosage, which is much greater compared to what is required in distal renal tubular acidosis (dRTA), depends on the extent to which the tubular reabsorption process is impaired [5, 6]. Normally the initial dose of bicarbonate necessary prescribed is 10 to 15 mEq/kg per day, given in divided doses, trying to overcome urinary bicarbonate losses and raise serum levels. If blood tests demonstrate persistent metabolic acidosis with low levels of HCO3-, the dose of alkali must be progressively increased. Furthermore, the urinary loss of bicarbonate leads to urinary potassium loss as well because increased sodium bicarbonate and water delivery to the distal tubule stimulate potassium secretion. Therefore, an empirically determined fraction of the alkali replacement must be given as a potassium salt.

Several preparations of oral bicarbonates can be prescribed, depending on the age of the patient and the amount of bicarbonates required: oral formulations are available via tablets (325 or 650 mg tablets, mostly used in adult patients), powder (baking soda, not routinely used, except in poor settings) and solutions (preferable for pediatric patients) [7]. However, in children it may be impractical to prescribe sodium bicarbonate solutions because of the high quantity that would be required to provide adequate levels of serum HCO3-. Moreover, in case of severe pRTA, as in the report described, bicarbonates renal loss may be massive, so that a continuous supplementation of alkali rather than boluses may be required. The overall alkali dose requirement could be reduced by diminishing the bicarbonate wasting with thiazide diuretics, that enhances bicarbonate reabsorption in the proximal tubule by reducing extracellular volume. However, thiazide diuretics also increase urine potassium losses, worsening the hypokalemia: therefore, the use of these drugs is impractical because it would be necessary to introduce a potassium-sparing diuretic such as amiloride or spironolactone, that further increases the drug burden [8].

Based on these considerations, the Mitochondrial Medicine Society recommends the placement of a percutaneous gastrostomy when a large amount of alkali is necessary to obtain a normalization of acid-base equilibrium [9, 10]. However, we are not aware of any report highlighting in children how dramatically this approach, coupled with an enteral nocturnal administration, can change the patient’s and family quality of life. Moreover, precise guidelines on how to the set the alkali supplementation via PEG throughout the day are currently lacking.

This report suggests that the combination of a nocturnal continuous enteral administration of alkali, combined with diurnal boluses, may represent a convenient solution. Firstly, it reduces the fluctuation of bicarbonates serum levels, allowing persistent and appropriate levels of HCO3-. Secondly, it improves quality of life in children, who no longer need to assume large amounts of oral unpalatable solutions many times a day. Furthermore, the nocturnal enteral administration allows a normal sleep cycle, avoiding night awakening to assume bicarbonate, which is almost mandatory at some point in conditions like KSS (Table 4).

Since its introduction in 1980, PEG has gained world-wide acceptance as a safe technique for providing enteral feeding and enteral therapy administration in patients with difficult or poor oral intake [11]. It is considered a minimally invasive procedure to ensure adequate source for enteral nutrition and drug intake in adults and children affected by chronic conditions. Complications of PEG are rare and most of them are considered minor as can be prevented with appropriated nursing cares [12]: granuloma formation around the gastrostomy, local wound infection, tube blockage and tube dislodgment are the most common problems observed. Although PEG needs daily care and periodic replacement of the gastrostomy button (every 3–6 months), it is usually well-tolerated.

We believe that benefits obtained by the percutaneous gastrostomy overcome the risks related to the PEG placement, and that the enteral administration of bicarbonates should be considered not only in mitochondrial disorders, but also in other clinical conditions where metabolic acidosis due to renal bicarbonate loss cannot be controlled by oral alkali implementation.

**Table 4:** Advantages in the administration of alkali via PEG

Advantages in the administration of alkali via PEG
- Improved quality of life • No limits in diurnal activities nor sleep interruptions to assume oral bicarbonate • Avoidance of aversion to alkali oral assumption
- Possibility to administer large amount of alkali reaching adequate HCO3- levels
- Reduced fluctuation of bicarbonates serum levels through nocturnal continuous administration

## Data Availability

All data generated or analyzed during this study are included in this published article and its supplementary information files.

## Abbreviations

MDs: mitochondrial diseases
MELAS: mitochondrial encephalomyopathy, lactic acidosis and stroke-like episodes
KSS: Kearns-Sayre syndrome
PEG: percutaneous gastrostomy
pRTA: proximal renal tubular acidosis
dRTA: distal renal tubular acidosis
